# Application of Educational Psychology Based on Improved SPBO Optimization Algorithm in English Learning

**DOI:** 10.3389/fpsyg.2022.949568

**Published:** 2022-07-29

**Authors:** Yingying Peng

**Affiliations:** School of Foreign Languages, Hubei University, Wuhan, China

**Keywords:** improve SPOB optimization algorithm, educational psychology, English learning, English teaching percentage value evaluation, emotional incentives

## Abstract

It is an inevitable process of current social development to apply the motivational theory of educational psychology in the field of English teaching. The current method is to start with the introduction of new language teaching projects by teachers, and then use excellent training to make students master the knowledge they have learned. The flaw is that such teaching is simplistic in the present. In order to solve these problems, this paper proposes an improved SPOB optimization algorithm, aiming to study the application of motivation theory in educational psychology to current English teaching. By using the formula definition for the excellent and poor students in the improved SPBO optimization algorithm and the criterion function in the cluster analysis, the application process of motivational design model in oral English teaching is explored through the application of SPBO algorithm. And through the investigation and analysis of the experimental process of the application of incentive design model in oral English teaching, the results showed that 77.2% of teachers chose interest incentives, 34.8% of teachers chose cooperation-competition incentives, and 32.6% of teachers chose emotional incentives.

## Introduction

Related research shows that motivation is not only the source of foreign language learning, but also the continuous driving force in the language learning process. Compared with language ability, motivation plays a greater role in foreign language learning. With the entry into the 21st century, English has played a key role in various fields. Therefore, learning English has become a basic requirement for students in today's society.

First, this study expanded the field of motivation research, integrated the research results of motivation in educational psychology, social psychology, performance technology and foreign language teaching, and expounded motivation theory from multiple perspectives and levels. Secondly, this study combined the practice of specific oral language textbook design, development and implementation, and used methods such as literature synthesis, questionnaire survey and experimental comparison to enrich the research methods in this field. Third, this study used educational technology as a bridge to explore how educational technology provided strong support for incentive design. Finally, this topic explored the practical operation of incentive design in oral English teaching, which had great practical guiding significance for the current teaching and training of various types of oral English.

Combining the practice of designing, developing and implementing multi-media oral English teaching materials, this paper attempts to integrate the motivational design model into the whole process of oral English teaching design with multi-media as the carrier, so as to summarize a relatively complete motivational design that can be used to guide teaching. This kind of exploration can have certain guidance and reference value for solving the motivation problem of English teaching clock and for the current booming English teaching and training.

## Related Work

Educational psychology is used to study people's learning in educational settings and has important implications for instructional interventions and pedagogical psychology, even including the social psychology of organizations. The research applications of educational psychology are as follows. The main focus of Chelghoum A 's research was to support students' self-regulation (Chelghoum, 2017). Bailey JH studied the psychology of education that underlay the categories of learning that occurred in clinical settings, and believed that understanding this was critical to creating opportunities for learners to activate their knowledge base at the precise time of appropriate application (Bailey and Rutledge, 2017). Priantini (2021) aimed to study the implementation of learning in educational psychology courses, which were often boring and low in learning outcomes, and the data collection tool for the study was an assessment form for expert testing and student testing. Rashid et al. (2021) proposed that in today's complex educational systems, educational psychologists work with educators, administrators, teachers, and students needed to learn more about how to help education. Peng analysis was used to compare learning performance, learning motivation, and self-regulated learning across educational stages, ages, and programming experiences. The results showed no difference in learning performance between the two educational settings (Peng and Bai, 2020). The knowledge of educational psychology is not often reused in the current society. Many experiments first only exists in the theoretical stage and cannot carry out practical research. However, the above-mentioned research is only at the theoretical stage, and the practical effect is not very good.

SPBO, a meta-heuristic algorithm recently proposed that simulates the psychology of students to improve their performance in all subjects to secure the best spot in the class. The initial population of the SPBOA study is similar to a class of students. Each group or student consists of different variables that correspond to the various subjects they have available. Students are recognized for their efforts if their overall performance on the exam improves. Pal and Mukherjee (2021) designed a global MPPT controller for the psychological optimization of students to improve the overall performance of the 4S and 3S configurations of the photovoltaic array. Dash and Mishra (2021) introduced the first engineering application of a recently proposed metaheuristic algorithm, an optimization algorithm based on student psychology, which simulated the psychology of students in a class to continuously improve their class performance and become the best students. Sasmito proposed an efficient optimization algorithm called optimization based on student psychology to solve the bi-objective permutation flow shop scheduling problem. The SPBO algorithm did not require any tuning parameters, which made computational experiments simpler. The original SPBO classified students in relation to their efforts to improve their performance (Karthika et al., 2020; Sasmito and Pratiwi, 2021). However, the current research on English teaching in educational psychology under the SPOB algorithm still does not get rid of the thinking and methods based on traditional English teaching, and also lacks in-depth analysis and discussion of the functionality of the Internet of Things.

## Optimization Algorithm Based on Student Psychology

### Optimization of Artificial Intelligence Classifiers

In order to improve the performance of artificial intelligence classifiers, SPBOA is used to automatically adjust the variables of each artificial intelligence. For artificial neural networks, the learning rate and momentum rate are used as variables (Navarro-Guzmán and Aragón-Mendizábal, 2021). This is due to the fact that the learning rate affects the scale of the respective adjustments or small, while the momentum constantly speeds up the training process. To optimize the performance of KNN, the number of nearest neighbors k is adjusted to specify the number of nearest neighbors to classify each point when predicting, while keeping the adjustment similar to NB (Sun et al., 2021). The variables of each AI classifier optimized by SPBOA are shown in Table 1.

**Table 1:** Variables for each Al classifier used for SPBOA optimization.

**Al classifier**	**Variable**	**Range**
ANN	Learning rate	0.01–1
	Momentum constant	0.01–1
SVM	Sigma, o	0.01–1
	Box Constraint, c	0.01–1
NB	Holdout	0.1–1
	Width	0.1–1
KNN	Number of nearest neighbor k	1–20
	Holdout	0.1–1

The fitness function that SPBOA uses to optimize AI performance is the minimization of the fault determination error or the maximization of the fault determination accuracy given by the function as:


(1) $$\begin{array}{l} Fitness\;function=\min\left(100\%-Accuracy\%\right) \end{array}$$

Among them, Accuracy% is calculated by the formula.

The Student Psychology-Based Optimization Algorithm (SPBOA) is a newly introduced meta-heuristic algorithm developed based on student psychology, which attempts to achieve top grades and become top students by improving academic performance.

(1) Best student

The best student is the one with the highest overall score in the exam, who will make every effort to maintain the rank by achieving the highest score in the class. To keep the position, more effort need to be put in each subject than others (Li et al., 2021). Balance can be used to express the progress of the best students as follows:


(2) $$\begin{array}{l} X_{bestnew}=X_{best}+{\left(-1\right)}^{k}rand\left(X_{best}-X_{j}\right) \end{array}$$

XBest is the grade of the best student and *X*_*j*_ is the grade obtained by the jth student in a randomly chosen subject, k is a parameter randomly chosen to be 1 or 2, and rand is a number between 0 and 1.

(2) Good students

A good student puts more effort into the favorite subjects and overall performance improvements. Due to the psychological diversity of students, good students are randomly selected. In order to get the highest score in the test to become the best student, some students try to meet or exceed the best student's efforts (Schalkwyk, 2021). The following formula can be used to represent this student category:


(3) $$\begin{array}{l} X_{newi}=X_{best}+rand\left(X_{best}-X_{i}\right) \end{array}$$

At the same time, some students try to put more effort into their studies and mimic the efforts of the best students. The following formula can be used to represent this student type:


(4) $$\begin{array}{l} X_{newi}=X+rand\left(X_{best}-X_{i}\right)+rand \end{array}$$

X means the average grade of the class in a particular subject, i is the grade achieved by the ith student in a particular subject.

(3) Average number of students

Since students' effort is determined by their interest in the subjects offered to them, if they are not too interested in the subjects, average effort is paid. Of the average effort placed in that subject, other subjects will put in more effort to improve their overall grade (Schwartz et al., 2020). This group of students can be described as the average student in each subject. The selection of this student is random and depends on the psychology of each student. The following formula can be used to represent the performance of this group of students:


(5) $$\begin{array}{l} X_{newi}=X_{i}+rand\left(X_{mean}-X_{i}\right) \end{array}$$

X means the average grade of the class in a particular subject, i is the grade achieved by the ith student.

(4) Students who try to improve their learning at random

Some students try to improve grades by making different efforts in different subjects at different times. This category of students attempts to put a random effort into each subject to improve their overall test scores. The following can be used to indicate student performance in this category:


(6) $$\begin{array}{l} X_{newi}=X_{min}+rand\left(X_{mean}-X_{min}\right) \end{array}$$

### SPBOA Algorithm

(1) Optimization algorithm based on student psychology

The overall algorithm of SPBOA incorporates the above four types of student psychology. The initial population of the SPBOA study is similar to a class of students (Li et al., 2022). Each group or student consists of different variables that correspond to the various subjects they have available. Students are recognized for their efforts if their overall performance on the exam improves. Changes in variables are also accepted when the fitness of the population is better. This algorithm takes some students into account, and the overall algorithm is shown in Figure 1.

**Figure 1:** Overall algorithm flow chart.

As can be seen from the above, Figure 1 contains the above four types of student psychology. Students' classroom performance is often influenced by several factors such as students' interest, efficiency, and ability, making it a random process. To simulate this, this paper proposes a normal distribution characterized by a mean or mean (u) and a distribution (o) that unambiguously matches the stochastic process of student performance in the class. Since the psychology of individual students in exams is different from other students, it is also recommended to have similar psychology for different groups of students (Ucha et al., 2021).

Different groups of students tend to have different psychology for improving performance. The student with the highest grade in the exam is considered the best student. It may be necessary for a top student to perform better than any other student on a test. Therefore, the improvement in performance can be expressed as the following formula:


(7) $$\begin{array}{l} p_{ij}^{k+1}=p_{best,ij}^{k}+{\left(-1\right)}^{a}*rand*\left(p_{best,ij}^{k}-p_{rj}^{k}\right) \end{array}$$

(8) $$\begin{array}{l} p_{ij}^{k+1}=p_{best,ij}^{k}+rand*\left(p_{best,ij}^{k}-p_{ij}^{k}\right) \end{array}$$

(9) $$\begin{array}{l} p_{ij}^{k+1}=p+\left[rand*\left(p_{best}^{k}-p_{ij}^{k}\right)\right]+\left[rand*\left(p_{ij}^{k}-p_{average}^{k}\right)\right] \end{array}$$

It can be seen from the Formula 7–9 that $p_{average}^{k}$ is the average grade of students in the class in *k*^*th*^ iteration. In the case of the average student, such as the student trying to put in an average effort, it can be expressed by the Formula 10:


(10) $$\begin{array}{l} p_{ij}^{k+1}=p_{\min,j}+\left[rand*\left(p_{\max,j}-p_{\min,j}\right)\right] \end{array}$$

Furthermore, it outperforms other state-of-the-art meta-heuristics in solving the standard benchmark functions claimed in the formulas. Hence, it makes it a strong contender for recent state-of-the-art metaheuristics that can be used to solve different optimization problems (Ahmadi and Dehghani, 2022).

In this paper, the SPBO algorithm is used in the general model part of the teaching system design, and its formula for good and bad is used to summarize a teaching system with strong versatility. And then its randomness and data analysis capabilities are used to help the investigation of the results.

(2) Criterion function in cluster analysis based on SPOB algorithm

When a specific function is used to evaluate the criterion of the pros and cons of the strategy adopted by the system, it is called a criterion function. The type of actual problem and the value of the criterion function depend on the strategy adopted by the decision maker. If a certain strategy can make the criterion function reach the optimal value, this strategy is called the optimal strategy of this criterion.

The criterion function is defined as:


(11) $$\begin{array}{l} G_{l}=\sum p_{j}s_{j} \end{array}$$

(12) $$\begin{array}{l} s=\frac{2}{n_{j}\left(n-1\right)}\underset{x\in x_{i}}{\sum }\underset{x\in x_{j}}{\sum }{\left\|x-x^{\prime }\right\|}^{2} \end{array}$$

*p*_*j*_ is the weight and *s*_*j*_ is the average squared distance between the data within the class.

(3) Error sum of squares criterion function

The criterion function is expressed as:


(13) $$\begin{array}{l} G_{c}=\overset{K}{\underset{j=1}{\sum }}\underset{u\in U_{j}}{\sum }d\left(x_{u},c_{j}\right) \end{array}$$

(14) $$\begin{array}{l} c_{j}=\frac{1}{N_{j}}\sum x_{u} \end{array}$$

In the formula, K is the number of classes, *U*_*j*_ is the sample in class j, *x*_*u*_ is the position vector of the sample in class j, *c*_*j*_ is the center point position vector in class j, and *N*_*j*_ is the number of samples in class j.

(4) Inter-class distance and criterion function

The inter-class distance and the criterion function reflect the distance between the various classes, which represent the degree of separability between the classes. The larger the value of the function, the better the clustering result. The two existing inter-class distance and criterion functions are defined as follows:

Inter-class distance and function:


(15) $$\begin{array}{l} G=\overset{K}{\underset{j=1}{\sum }}\left[{\left(c_{j}-X\right)}^{T}\left(c_{j}-X\right)\right] \end{array}$$

Weighted inter-class distance and criterion function:


(16) $$\begin{array}{l} G_{2}=\overset{K}{\underset{j=1}{\sum }}\left[p_{j}{\left(c_{j}-X\right)}^{T}\left(c_{j}-X\right)\right] \end{array}$$

In the formula, *c*_*j*_ is the center point position vector of class j, X is the data in the data set, and *p*_*j*_ is the prior probability of class j.

(5) Overview of K-means clustering algorithm

The algorithm is an iterative algorithm. First, the distance between the sample object and the center point of each cluster is calculated, and then each sample is divided into the cluster domain closest to itself.

The criterion function of the algorithm is:


(17) $$\begin{array}{l} G={\overset{K}{\underset{j=1}{\sum }}\underset{u\in U_{j}}{\sum }\left(x_{u}-c_{j}\right)}^{2} \end{array}$$

(18) $$\begin{array}{l} c_{j}=\frac{1}{N_{j}}\underset{u\in U_{j}}{\sum }x_{u} \end{array}$$

In the formula, K is the number of classes, *U*_*j*_ is the sample in class j, *x*_*u*_ is the position vector of the sample in class j, *c*_*j*_ is the position vector of the center point of class j, and *N*_*j*_ is the number of samples in class j.

### Core Idea of K-means Algorithm Based on SPBO Algorithm

The K-means algorithm is to divide a data set containing n data into k classes, and to minimize the value of the criterion function that satisfies the clustering. The distance from each data to each cluster center is calculated, and the data is divided into the classes closest to them. After all data processing is complete, the cluster center is recalculated using the Formula 19:


(19) $$\begin{array}{l} c_{j}=\frac{1}{n}\underset{x\in C_{j}}{\sum }x \end{array}$$

Clustering is to make the similarity between data in the same class as high as possible, and the similarity between data in different classes as small as possible (Elhadary, 2021). The similarity measure of the K-means algorithm uses the Euclidean distance. The minimum distance principle is used to divide the attribution of the data. The convergence of the objective function (such as the criterion function) is the ultimate goal of the algorithm. The objective function of the K-means algorithm is the error sum of squares function (Gu et al., 2021). As shown in the Formula 20:


(20) $$\begin{array}{l} J=\overset{k}{\underset{j=1}{\sum }}\overset{n}{\underset{i=1}{\sum }}d_{i,j}\left(x_{i},c_{j}\right) \end{array}$$

The termination condition of the algorithm is often that there is no change in the adjacent two cluster centers, the change of the objective function value is within a certain threshold, or the number of running iterations is greater than the set maximum number of iterations. The K-means algorithm is actually looking for the K partitions with the smallest objective function.

From the above, it can be seen that the improved SPBO algorithm and the cluster analysis method are two of the current advanced and popular algorithms, using the accuracy of its excellent difference formula and criterion function, which can provide help for the following researches on motivation theory in oral English teaching and English teaching.

## Application Design of Motivational Theory in Educational Psychology in Oral English Teaching

### Educational Technology—Bridge Between Communication Motivation Theory and Oral Language Teaching Practice

This paper mainly discussed how to carry out effective incentive design in oral English teaching. Therefore, researches involving three fields of educational technology, motivation (incentive) theory, and oral language teaching are shown in Figure 2.

**Figure 2:** Relationship between educational technology, motivation theory, and oral language teaching.

In the figure, educational technology, as a bridge to communicate oral English teaching and motivation theory, can provide strong theoretical and technical support for the motivation design in oral English teaching (Elena and Prokopenko, 2019).

(1) The process definition of educational technology

In educational technology, problem solving takes the form of designing or selecting and using learning resources to facilitate learning. The process of analyzing the problem and designing, implementing and evaluating the method to solve the problem is called the educational development function, which includes research and theory, design, production, evaluation and selection, supply, utilization and promotion (Hong et al., 2019a). The process of directing or coordinating one or more of these functions becomes an educational management function, which includes organizational management and personnel management. The operating model of its technical field is shown in Figure 3.

**Figure 3:** Operational model flowchart.

It can be seen from Figure 3, educational technology consists of four aspects: learners, learning resources, educational development functions and educational management functions. First, it is the process of applying a systems approach to analyzing and solving human learning problems, and then relying on the development and utilization of all learning resources to achieve goals.

(2) Requirements for motivation in teaching theory and practice

As one of the three theoretical cornerstones of educational technology, learning theory mainly explores the nature of human learning and its formation mechanism. In the process of discussing learning rules, three schools have been formed: behavioral learning theory, cognitive learning theory and constructive learning theory. They explain the nature and process of human learning knowledge and skills from different perspectives, and give different guiding principles to specific teaching practices (Koroleva, 2021). As shown in Figure 4.

**Figure 4:** Flowchart of the specific tasks of the teacher's role.

Figure 4 embodies the main motivational ideas and strategies in the motivational design model and the super-incentive model. Among them, R1, R3 and C1 in the figure emphasize the incentive strategy of “attracting the learner's attention”; X1, R2 emphasize the incentive strategy of “establishing the connection between learning and the learner's needs and their original learning experience”; X2, C3 emphasize the incentive strategy of “giving necessary learning support and improving self-confidence in learning”; X3 emphasizes the incentive strategy of “providing timely feedback and improving learner satisfaction”; and C2 embodies the incentive thought of “creating a stimulating learning environment” (Abdullah et al., 2021).

The ARCS model focuses on the selection and combination of incentive strategies, while the time continuum model focuses on the order in which incentive strategies are implemented. The model, framed in time, summarizes six categories of factors that influence motivation: attitudes, needs, stimuli, emotions, abilities, and reinforcement (Hong et al., 2019b). Furthermore, the model divides the teaching process into three stages (beginning, progressing, ending) and proposes appropriate motivational strategies for each stage. As shown in Table 2:

**Table 2:** Application of time continuous model in specific teaching.

**Teaching process**	**Main motive factor**	**Incentive strategy**
Start	Attitude and need	Creating a positive, safe, and interesting teaching environment.
Process	Stimulating and emotion	Change the content and form of teaching activities to stimulate learners' participation enthusiasm. Through the “Solving Issues”, “Role Playing” and other teaching forms allow learners' participation and reactions to the core part of learning.
Finish	Ability and enhancement	Continuous feedback on learners' learning.

### Incentive Design of Multi-media Oral English Teaching

(1) General model of teaching system design

Instructional design, or instructional system design, is a concrete and operational procedure for implementing an instructional system approach. In the process of teaching system design, many educational technology scholars have put forward many theoretical models with considerable reference value. Although there are many different teaching system design models, a general model of teaching system design with strong generality can be summarized from the common characteristics of these models (Ahmed et al., 2021). This paper will extract the basic components of instructional design from various theoretical models, and construct a general model of instructional system design, as shown in Figure 5.

**Figure 5:** General model of instructional system design.

The general model of instructional design divides instructional system design into five stages: analysis, design, development, implementation, and testing, and summarizes the tasks of each stage:

(1) Analysis stage:

The “why and what to teach” process is defined, the nature of the learning task and where and when to teach are determined.

(2) Design phase:

It is the process of defining “how to teach”. The main tasks of this stage includes: making a specific and clear description of the learning objectives; clarifying the final behavioral state that should be achieved after learning.

(3) Development stage:

The process of writing and producing textbooks. The main tasks of this stage are: selecting and adapting existing teaching materials or writing new teaching materials, including textbooks, workbooks, diagrams, pictures, animations, and training instruction manuals, etc.; developing the hardware of the teaching media system; developing software for the operating system; courseware development and production; testing and verification of the interactive performance between teachers, learners and teaching systems.

(4) Implementation stage:

The process of implementing an instructional design program. The main tasks of this stage are: recruiting learners who meet the admission requirements; teaching arrangements, including teaching venues and teaching organization forms, etc.; carrying out teaching work; maintaining normal teaching order; creating a good learning environment; and ensuring teaching facilities, equipment and The supply of teaching materials; monitoring the teaching progress, timely diagnosis of teaching problems and taking corresponding remedial measures.

(5) Inspection and feedback:

Formative assessments should be conducted in the teaching process. It refers to the external evaluation standards of the teaching system and the evaluation methods of related jobs to test the reliability and validity of the teaching behavior evaluation standards, and provides feedback for the improvement and maintenance of the teaching system.

(2) Integration of motivational design model and oral English teaching design

Combined with oral English teaching, this paper attempts to integrate the specific application of the incentive design model in each stage of teaching design. The purpose is to propose an exploratory reference frame for how to carry out effective incentive design in oral English teaching. As shown in Figure 6.

**Figure 6:** Integration of models.

Figure 6 is the five stages of the instructional design process, namely analysis, design, development, implementation and evaluation. The vertical axis is the four types of motivational factors in Keller's motivational design model, namely attention, relevance, self-confidence and satisfaction. The “inspection and feedback” at the bottom of the model refers to the formative evaluation in the process of instructional design, its purpose is to test, revise and improve the work of each stage of instructional design, so as to form the most suitable teaching for learners. The arrows in the figure represent the two-way information flow between the stages, and its role is to provide timely feedback for the improvement and maintenance of the system. Another purpose of the arrow is to illustrate that the teaching system design is a dynamic process of continuous revision and improvement.

## Results of Motivation Theory in English Teaching

### User's Evaluation of Incentive Theory

This paper used the Textbook Motivation Questionnaire and the Curriculum Interest Questionnaire to measure all learners' responses to the motivational design effect of this set of textbooks and their motivational status in the oral classroom. It used the criterion function in the cluster analysis part based on the SPBO algorithm to construct the textbook incentive questionnaire and the curriculum interest questionnaire. The Cronbach's alpha coefficients of these two measurement tools were above 0.8, indicating that they had high internal reliability and could be used to evaluate the effect of oral language teaching incentive design.

The Textbook Motivational Questionnaire (IMMS) designed 36 questions around four motivational factors: attention, relevance, confidence and satisfaction. According to the subject's possible opinion on the description of the item, the evaluation was divided into five levels: disagree, slightly agree, partially agree, basically agree and fully agree, which were expressed in turn from A to E. For most of the questions in the questionnaire, A–E corresponds to the score The score is 1–5 points, and for a few items with negative responses (shown in italics), the corresponding points of A–E are 5–1 points. According to this standard, the score statistics were carried out, and the total score of all items was the lowest. Divided into 36 points, the highest score was 180 points, the middle value was 108 points.

First the total score was divided into five fractional segments with the same interval: 0–36, 36–72, 72–108, 108–144, 144–180. These five score segments corresponded to five different grades: very poor, poor, average, good, and good, as shown in Table 3.

**Table 3:** The distribution of the total score of the textbook incentive questionnaire.

**Evaluation**	**Fraction**	**Number of responds**	**Percentage**
Very bad	0–3	0	0
Difference	36–72	0	0
Generally	72–108	0	0
Better	108–144	17	56.67%
Very good	144–180	13	43.33%

The data in the table shows that all learners believe that the motivational design of the textbook has generally good or good effects. Secondly, the score of each item is counted, and it is found that most learners believe that the textbook has achieved good results in the incentive design of the four types of factors, among which the incentive design of the “attention” factor is particularly prominent, as shown in Figure 7.

**Figure 7:** Statistical chart of survey analysis of incentive design.

From Figure 7, it can be seen that the 30 subjects' evaluations of the motivational design effects of the textbook in terms of “attention”, “relevance”, “confidence” and “satisfaction” are all at the middle and upper level, with the highest point being 0.820. The lowest point is 0.776, and the scoring rate is above 0.500. The highest point is the “attention” item, which shows that the learners think that the textbook does the best job in attracting and maintaining attention, which proves that the textbook can stimulate and maintain the interest in learning oral language. The lowest point is the “self-confidence” item, and the score of six questions in this item is lower than four points, which shows that the motivational design of the textbook in cultivating and enhancing the self-confidence of learners is relatively insufficient and needs to be improved.

The Curriculum Interest Inventory (CIS) was designed to measure learners' motivation in oral classroom teaching organized by teachers. The scale had 34 questions designed around four motivational factors of attention, relevance, self-confidence and satisfaction, and its scoring method was the same as that of the Textbook Motivational Questionnaire (IMMS). According to this standard, score statistics were carried out. The lowest score of all items was 34 points, the highest score was 170 points, and the middle value was 102 points. First, the total score of the 30 subjects was divided into five score segments according to the same group distance: 0–34, 34–68, 68–102, 102–136, 136–170. These five score segments corresponded to five different grades: very poor, poor, average, good, and great. The data in the table shows that all learners believe that their interest in oral language learning is better stimulated and maintained in the classroom. They also gave good evaluations to teachers' motivational performance as shown in Table 4.

**Table 4:** Statistics of the total score distribution of the course interest questionnaire.

**Evaluation**	**Fraction**	**Number of responds**	**Percentage**
Very bad	0–34	0	0
Difference	34–68	0	0
Generally	68–102	0	0
Better	102–136	P	60.00%
It is good	136–170	12	40.00%

Secondly, the statistics of the scores of each item were carried out, and it was found that most learners believed that teachers and oral textbooks played a good role in the incentive design of the four types of factors, as shown in Figure 8.

**Figure 8:** Course interest survey statistics.

### Investigation on the Current Situation of the Implementation of Classroom Teaching Incentive Theory for Primary School English Teachers

(1) Teachers' attention to student motivation in different course types.

A total of 94 primary school English teachers in a city were surveyed. Ninety-four questionnaires were issued and 92 were returned. Using SPBO algorithm to organize and analyze the data, and the survey results were obtained. Combined with the subjective part of the questionnaire, the questionnaire was deeply analyzed to find out the problems.

In different course types, teachers paid different attention to the implementation of student motivation. In new teaching, teachers paid more attention to the motivation of students' interest (70.7%), and cooperation-competition incentives (43.5%); in review classes, 50% of teachers were more concerned about feedback-evaluation incentives for students, and cooperation-competition incentives (43.5%); the cooperation-competition incentives of students were the most important, accounting for 69.6% of the total ratio, followed by the incentives for students' interests (26.1%); in the comprehensive activity class, teachers were most concerned about the following two aspects, one was the incentive of cooperation-competition of students (46.7%), and the incentive of interest with students (44.6%). From the survey data, it could be seen that the proportion of teachers implementing cooperation-competition incentives for students was relatively stable, and they all occupied a large share. It could be seen that in the process of students' English learning, the current primary school English teachers paid close attention to the motivation of students' cooperation-competition. In any course type, the frequency of teachers' use was high enough to show the popularity of cooperative-competitive incentive strategies. Secondly, it could be seen that in different course types, teachers' attention to motivation was different, for example, interest incentives in new classes, feedback-evaluation incentives in review classes, cooperation-competition incentives in practice classes and comprehensive activity classes. Through such data, the current teacher's curriculum design and implementation is as shown in Figure 9.

(2) Attention to incentives in each course link

**Figure 9:** Classroom teaching incentives in various types of courses. **(A)** Classroom teaching incentives for new classes. **(B)** Classroom teaching incentives for review classes. **(C)** Classroom teaching incentives for drills.

Here is the focus on motivation in each course segment. The survey data showed that the current primary school English teachers paid different attention to incentives in each link, as shown in Figure 10.

**Figure 10:** Statistical chart of the influence of teaching incentives in various links in the classroom. **(A)** Revision link teaching incentive statistics. **(B)** Presentation link teaching incentive statistics.

It can be seen from Figure 10 that in the revision link of the English classroom, teachers paid the most attention to the motivation of students' feedback-evaluation; in the presentation link, teachers paid the most attention to the motivation of students' cooperation-competition and goals; these data further verified the above teachers' attention to different aspects of students' motivation in various lesson types. It can be seen that the data was known, which showed that teachers paid more attention to interests and goals in the presentation of knowledge introduction words. In the review of classroom knowledge, the link focused on feedback-evaluation, and in the practice, it focused more on the incentive of cooperation-competition.

## Conclusions

Based on the improved SPOB optimization algorithm, this paper explored and studied the application of educational psychology in English teaching. Using the SPOB algorithm and the cluster analysis algorithm based on the SPOB algorithm, it explored, analyzed and motivated English teaching from the part of motivation theory in educational psychology, in short, it was to stimulate and encourage, mobilize people's enthusiasm, initiative and creativity; their internal and external motivation were stimulated, maintained and enhanced, their behavior was induced, making them realize their potential, and achieving the goals pursued the process of effort. However, the current motivation theory is still in its infancy in the field of English teaching, and has not been well-publicized and evaluated. So in the future, it is necessary to start from many aspects, not only English speaking teaching, situational dialogue, article translation, etc., and other teaching parts which should use motivation theory to stimulate students' interest in English.

## Data Availability Statement

The original contributions presented in the study are included in the article/supplementary material, further inquiries can be directed to the corresponding author/s.

## Author Contributions

YP: writing—original draft preparation and editing data curation and supervision. The author confirms being the sole contributor of this work and has approved it for publication.

## Conflict of Interest

The author declares that the research was conducted in the absence of any commercial or financial relationships that could be construed as a potential conflict of interest.

## Publisher's Note

All claims expressed in this article are solely those of the authors and do not necessarily represent those of their affiliated organizations, or those of the publisher, the editors and the reviewers. Any product that may be evaluated in this article, or claim that may be made by its manufacturer, is not guaranteed or endorsed by the publisher.
